# Prognostic Value of MUC16 Mutation and Its Correlation with Immunity in Hepatocellular Carcinoma Patients

This article has been retracted.

**DOI:** 10.1155/2022/3478861

**Published:** 2022-08-18

**Authors:** Bing Liu, Zhicheng Dong, Yingzhi Lu, Jianhua Ma, Zhaoming Ma, Hongwei Wang

**Affiliations:** ^1^Department of Radiotherapy, The Second People's Hospital of Lianyungang (Lianyungang Cancer Hospital), Lianyungang, China; ^2^Oncology Department, The Second People's Hospital of Lianyungang (Lianyungang Cancer Hospital), Lianyungang, China

## Abstract

**Objective:**

Identifying gene mutation signatures will enable a better understanding for the occurrence, development, and prognosis of hepatocellular carcinoma (HCC) and provide some potential biomarkers for clinical practice. This study investigated the mutated genes in HCC patients and assessed their relationship with tumor mutation burden (TMB) and prognosis.

**Methods:**

The somatic mutation annotation format (MAF) document, mRNA expression matrix, and clinical information of HCC patients were obtained from the International Cancer Genome Consortium (ICGC) and the Cancer Genome Atlas (TCGA) database. The differences of TMB between the mutant type and the wild-type genes were detected using the Mann–Whitney *U* test. The link of gene mutations with prognosis was explored by the Kaplan–Meier analysis. The proportion of 22 immune cells' composition was measured using CIBERSORT algorithm.

**Results:**

The two databases screened 16 common mutated genes, which included TP53, TTN, LRP1B, ZFHX4, MUC16, OBSCN, CSMD3, FLG, CSMD1, SYNE1, SPTA1, USH2A, KMT2C, PCLO, HMCN1, and FAT3. After a series of analysis, MUC16 mutation was found to be highly correlated with TMB and was regarded as an independent factor predicting HCC. Furthermore, gene set enrichment analysis (GSEA) indicated that the MUC16 mutation was significantly involved in HCC cell metabolism.

**Conclusions:**

MUC16 mutation seems to be a valuable potential biomarker for HCC development and its overall survival.

## 1. Introduction

According to estimated number in 2020 (worldwide, both sexes, all ages), liver cancer has become the third leading cause of cancer-related death with a higher incidence of 905, 677 patients [1, 2]. As the main subtype of liver cancer, hepatocellular carcinoma (HCC) accounts for 85–90% of all liver cancer subjects [3, 4]. HCC is usually diagnosed at an advanced stage with a 5-year overall survival rate of only 12% [5]. Traditional treatments for HCC, including hepatectomy, surgical resection, liver transplantation, chemotherapy, radiotherapy, and molecular targeted therapy [6], also lead to poor therapeutic outcomes [7]. Therefore, some effective and novel biomarkers are required to improve the prognosis of patients with HCC.

There are about 30,000 genes in human cells, and these genes act as the targets of numerous genetic mutation events that happen over the course of a human life [8]. Many gene mutations are served as prognostic biomarkers for cancers, such as tumor protein P53 (TP53), phosphatase and tensin homolog (PTEN), and RB transcriptional corepressor 1 (RB1) mutations in prostate cancer, and phosphatidylinositol-4,5-bisphosphate 3-kinase catalytic subunit alpha (PIK3CA), Erb-B2 Receptor Tyrosine Kinase 2 (ERBB2), and KRAS proto-oncogene and GTPase (KRAS) mutations in gastric cancer, as well as E1A binding protein P300 (EP300) in bladder cancer [9–11]. The progression of HCC involves many factors, including environmental exposure, somatic mutations, and transcriptional or epigenetic variations [12], among which, genetic mutations of several key genes (e.g., TP53, catenin beta 1 (CTNNB1), and telomerase reverse transcriptase (TERT)) have considerable relevance to the carcinogenesis and prognosis of HCC [13–15].

In this study, we collected somatic mutation data and transcriptome data in HCC patients from International Cancer Genome Consortium (ICGC) and the Cancer Genome Atlas (TCGA) cohorts. The shared mutant genes in two databases were screened, and the association of these gene mutations with TMB and prognosis was further investigated. The study indicated that MUC16 mutation was related to TMB and promoted anti-tumor immunity in HCC.

## 2. Materials and Methods

### 2.1. Data Resource

All the data used in this study were obtained from the publicly TCGA database (https://portal.gdc.cancer.gov/) and the International Cancer Genome Consortium (ICGC) (https://dcc.icgc.org/). The approval from a local ethics committee is not required since the TCGA and ICGC data are open to the public. Patients with complete clinical information, survival data, and complete gene mutation data were included. Somatic gene mutations for TCGA samples (*n* = 389) and ICGC (*n* = 105) were, respectively, analyzed.

### 2.2. Identification of Key Mutational Genes

The mutation annotation data of HCC were detected by VarScan software (v.2.3.7) and then visualized by the GenVisR package. The characteristics of mutation from the two cohorts were visualized using waterfall plot. The shared mutation genes between the two cohorts were identified using a Venn plot. To explore the prognostic significance of identified mutation genes, the survival analysis was conducted using the “survival” package. The overall survival analysis of genes in wild-type group and mutant group was implemented using the survival package. The mutational genes were eligible if they were significant in the survival analysis with *P* value < 0.05. Furthermore, we explored the association between the mutation genes and TMB. To calculate the TMB value of individual, the total number of mutations counted was divided by the exome size (38 Mb was treated as the estimate of the exome size) [16].

### 2.3. Gene Set Enrichment Analysis

Gene set enrichment analysis (GSEA) as a computational algorithm was used to determine whether a prior defined set of genes presents statistically significant differences between two different biological states [17]. GSEA was performed to seek signaling pathways involved in HCC patients between the mutant group and the wild group of identified genes and exhibited significant differences (*P* value<0.05) in the enrichment of MSigDB Collection (c2.cp.kegg.v7.1.symbols.gmt). The top 10 significant pathways in mutant group were visualized using the gg-plot R package. Gene sets with a nominal *P* value < 0.05 were considered statistically significant.

### 2.4. Immune Cell Infiltration

The CIBERSORT tool is widely employed in investigating the proportions of 22 subtypes, which are human immune cell types in the microenvironment. By using CIBERSORT algorithm, this study calculated the HCC individuals' data and obtained the relative proportion of 22 infiltrating immune cells. We uploaded the gene expression matrix data to CIBERSORT (https://cibersort.stanford.edu/index.php) and acquired the immune cell infiltration matrix. A correlation heatmap was plotted to view the correlation of 22 types of infiltrating immune cells. The difference in immune infiltration between mutant group and the wild group of identified genes in 22 types of immune cells was visualized using violin plots.

### 2.5. Statistical Analysis

All statistical analyses in this study were done using R (version 3.6.3; https://www.r-project.org/). Group comparisons were implemented for continuous variables between mutant genes and TMB using the Mann–Whitney *U* test. Kaplan–Meier survival analysis was used to estimate survival differences between mutant group and the wild group of identified genes. Univariate and multivariate Cox regression analyses were adapted for survival analysis of clinical variables of patients, including age, sex, grade, stage, TMB, and MUC16. A *P* value <0.05 was considered statistically significant.

## 3. Results

### 3.1. Mutated Genes in HCC

The identification of mutation characteristics is necessary for the exploration of HCC pathogenesis. As demonstrated in Figures 1(a) and 1(b), the details of the top 30 genes with frequent mutation in HCC patients from the TCGA and ICGC databases were displayed in waterfall plots. The Venn plot presented that the following 16 genes were overlapped in these two datasets, including TP53, TTN, LRP1B, ZFHX4, MUC16, OBSCN, CSMD3, FLG, CSMD1, SYNE1, SPTA1, USH2A, KMT2C, PCLO, HMCN1, and FAT3, which were analyzed subsequently (Figure 1(c), Table 1).

### 3.2. Identification of Prognosis-Related Mutated Genes

It was observed that all 16 genes (TP53, TTN, LRP1B, ZFHX4, MUC16, OBSCN, CSMD3, FLG, CSMD1, SYNE1, SPTA1, USH2A, KMT2C, PCLO, HMCN1, and FAT3) were significantly associated with higher TMB in patients with HCC (Figure 2). Further Kaplan–Meier analysis was carried out to investigate the relationship between mutant group and the wild group of identified genes associated with prognosis in HCC via TCGA cohort. It was revealed that a significant difference was detected only in the two genes (*P*=0.014for MUC16; *P*=0.033for FLG, Figure 3) between the two groups. Since MUC16 (the cancer antigen CA125) is the most commonly used serum biomarker in cancers [18,19], MUC16 was selected for the following analysis. The demographic characteristics of the HCC patients from TCGA cohort are presented in Table 2. We then performed the multivariate survival analysis of all variables (stage, age, and MUC16 mutation status) with *P* < 0.05 in univariate analysis by Cox proportional hazards analysis, and the result showed that age (HR = 1.65, 95%CI = 1.18–2.31; *P*=0.003), stage (HR = 2.18, 95%CI = 1.54–3.08; *P* < 0.001), and MUC16 mutation (HR = 0.64, 95%CI = 0.44–0.93; *P*=0.018) were independent prognostic factors in individuals with HCC (Table 3).

### 3.3. MUC16 Mutation GSEA

By separating the transcriptome data of HCC into MUC16 wild type and mutation groups, the abnormally expressed genes in HCC may be identified. The application of GSEA in TCGA cohort demonstrated that MUC16 mutation was involved in in cell cycle, metabolic process, and immune process, such as aminoacyl tRNA biosynthesis, base excision repair, cell cycle, cysteine and methionine metabolism, DNA replication, fructose and mannose metabolism, glycosylate and dicarboxylate metabolism, one carbon pool by folate, oocyte meiosis, pyrimidine metabolism, RNA degradation, spliceosome, steroid biosynthesis, terpenoid backbone biosynthesis, valine leucine, and isoleucine degradation (Figure 4).

### 3.4. The Relationship between Tumor Immune Cell Infiltration and MUC16 Mutation in HCC

With the help of CIBERSORT algorithm, the immune infiltration compositions of 22 types of immune cells in HCC were calculated. The relative percent of 22 immune cell infiltrations in HCC samples was visualized based on the TCGA cohort and is presented in Figure 5(a). Correlation heatmap of the 22 types of immune cells is displayed in Figure 5(b). A majority of immune cells were negatively correlated with each other. For example, M0 macrophages were negatively associated with CD8 T cell (*r* = −0.44); resting NK cells were negatively associated with activated NK cells (*r* = −0.39); resting mast cells were negatively associated with activated mast cells (*r* = −0.35); resting memory CD4T cells were adversely associated with CD8 T cells (*r* = −0.38). The differential expressional proportion of immune infiltration cells in the HCC tissues between wild and mutation types of MUC16 is displayed in Figure 5(c). It was revealed that regulatory T cells (*P* < 0.001), activated NK cells (*P*=0.015), monocytes (*P*=0.025), and resting mast cells (*P*=0.013) in wild type of MUC16 were significantly higher than those in mutation type of MUC16 (all*P* < 0.05). In contrast, the infiltration rates of resting NK cells were clearly upregulated in mutation type of MUC16 compared to that in wild type of MUC16 (*P*=0.004).

## 4. Discussion

HCC is a serious health concern worldwide with high morbidity and mortality. HCC presents clear molecular heterogeneity, including numerous somatic genome mutations [20]. However, to date, gene mutations associated with TMB and immune response in HCC are not entirely clear.

In this study, somatic mutation landscapes of HCC were described in 389 samples from the TCGA cohort and 105 Japanese samples from the ICGC cohort. Subsequently, 16 genes were frequently mutated in two databases. MUC16 ranked the third-highest mutation frequency, after TTN and TP53. Then, all of the 16 genes were associated with higher TMB, and survival analysis demonstrated that only MUC16 mutation group presented a better OS than the wild-type group. TMB indicates the accumulation of somatic mutations in cancers, and a high TMB promotes the exposure of more neoantigens, which is likely to induce a T-cell-dependent immune response [21]. Therefore, we considered that MUC16 mutation may strengthen immune response. Furthermore, cell cycle and metabolic signaling pathways were significantly enriched in patients with MUC16 mutation. Tumor-infiltrating immune cell analysis showed that patients with MUC16 mutations infiltrated more resting NK cells, which is consistent with immune cells and pathways that play an important role in the tumor microenvironment and promote immune responses [22,23]. These findings demonstrate that MUC16 has a certain research value in HCC.

MUC16 belongs to a type I transmembrane mucin that encodes cancer antigen 125 (CA-125) [24]. It was first descried almost 40 years ago and was found to be a transmembrane mucin 20 years later [25]. MUC16 is an essential membrane protein that sustains normal cell function and plays a role in the development of numerous cancers [26,27]. The expression of MUC16 is usually located in the cell membrane or scattered in bodily fluids as a soluble form [28]. A recent study revealed that MUC16 mutations are associated with a better OS in individuals with gastric cancer. One of possible mechanisms is that MUC16 mutations activate the p53 pathway and DNA repair pathway [24]. Previous studies in melanoma, colorectal cancer, and cervical cancer have demonstrated that individuals with high TMB scores show a favorable OS if treated with immune checkpoint inhibitors [29–32]. In our study, MUC16 mutation group presented higher TMB scores when compared to MUC16 wild-type group. Thus, it was possible that the MUC16 mutation group will benefit from immune checkpoint inhibitor treatment. Knockdown of MUC16 revealed the link between MUC16 and HCC cellular functions, demonstrating that tumor-derived MUC16 serves as a suppressor of the anti-tumor immune response [33]. MUC16 is a protein with a large molecular weight. The MUC16 gene covers many mutations in HCC derived from the TCGA portal [33]. Thus, we believe that such mutations may affect the structural stability of MUC16, which influences the expression of MUC16 protein.

Furthermore, regulatory T cells, activated NK cells, monocytes, and resting mast cells were more abundant in the wild type of MUC16 group, whereas resting NK cells were more abundant in the mutation type of MUC16 group. NK cells as an important component of innate immune system are labeled by releasing cytokines and cytolytic activity against target cells. It was demonstrated that NK cells can selectively kill cancer stem cells, which suggest that NK cell-based therapy can be used as an effective treatment to suppress cancer relapse and metastasis [34,35]. A majority of the genes in MUC16 mutation were enriched in various cancer-related pathways, such as cell cycle and metabolic process, which demonstrated the critical role of the MUC16 gene in HCC.

The main limitation in our study is that the conclusions were drawn from bioinformatics analysis mainly about the prognostic value of MUC16 mutation and its correlation with immunity in HCC patients. Further research would be performed with larger sample sizes for exploring the prognostic value of MUC16 and FLG mutation in a clinical cohort as time and funding permit. Moreover, the role of MUC16 expression in the progression and metastasis in HCC was required to be confirmed by experiments in future. Nevertheless, MUC16 mutation is frequently mutated in HCC, and its mutation is associated with elevated TMB and contributes to anti-tumor immunity, which can act as a biomarker to forecast immune response.

## Figures and Tables

**Figure 1:** Overview of frequently mutated genes in HCC. Mutational landscape of the top 30 frequently mutated genes in HCC in TCGA cohort (a) and ICGC cohort (b). (c) Venn diagram presents 16 frequently mutated genes shared by both databases.

**Figure 2:** Sixteen gene mutations are associated with TMB. Note: ^*∗*^*P* < 0.05; ^*∗∗∗*^*P* < 0.005.

**Figure 3:** Overall survival of individuals with HCC in wild type and mutation type of 16 gene mutations.

**Figure 4:** GSEA of the abnormally expressed genes in HCC in MUC16 mutation type.

**Figure 5:** The landscape of immune cell infiltration in HCC samples. (a) Bar charts of 22 types of immune cells in HCC samples. (b) Correlation matrix of 22 types of immune cell proportions. (c) Differential expression of 22 types of immune cells in HCC samples between wild type and mutation type of MUC16.

**Table 1:** The information of 16 frequently mutated genes.

Gene	Full name	Chromosome position	Gene ID	Ensembl
TP53	Tumor protein P53	17p13.1	7515	ENSG00000141510
TTN	Titin	2q31.2	7273	ENSG00000155657
LRP1B	LDL receptor related protein 1B	2q22.2	53353	ENSG00000168702
ZFHX4	Zinc finger homeobox 4	8q21.13	79776	ENSG00000091656
MUC16	Mucin 16, cell surface associated	19p13.2	94025	ENSG00000181143
OBSCN	Obscurin, cytoskeletal calmodulin and titin-interacting RhoGEF	1q42.13	84033	ENSG00000154358
CSMD3	CUB and Sushi multiple domains 3	8q23.3	114788	ENSG00000164796
FLG	Filaggrin	1q21.3	2312	ENSG00000143631
CSMD1	CUB and Sushi multiple domains 1	8p23.2	64478	ENSG00000183117
SYNE1	Spectrin repeat containing nuclear envelope protein 1	6q25.2	23345	ENSG00000131018
SPTA1	Spectrin alpha, erythrocytic 1	1q23.1	6708	ENSG00000163554
USH2A	Usherin	1q41	7399	ENSG00000042781
KMT2C	Lysine methyltransferase 2C	7q36.1	58508	ENSG00000055609
PCLO	Piccolo presynaptic cytomatrix protein	7q21.11	27445	ENSG00000186472
HMCN1	Hemicentin 1	1q25.3	83872	ENSG00000143341
FAT3	FAT atypical cadherin 3	11q14.3	120114	ENSG00000165323

**Table 2:** Demographic characteristics of the HCC patients from TCGA cohort.

Parameter	HCC patients
Age (years)	65.20 ± 10.59

Gender	
Male	251
Female	138

Grade	
G1	9
G2	138
G3	242

Stage	
I	51
II	126
III	175
IV	37

T stage	
T1	17
T2	80
T3	185
T4	107

M stage	
M0	348
M1	24
MX	17

N stage	
N0	122
N1	103
N2	79
N3	80
NX	5

**Table 3:** Univariate and multivariate overall survival analysis of HCC patients by the Cox proportional hazards.

Variables	Univariate		Multivariate	
	HR (95%CI)	*P*	HR (95%CI)	*P*
Age (≥65 vs. <65)	1.51 (1.08–2.10)	0.016	1.65 (1.18–2.31)	0.003
Gender (male vs. female)	1.01 (0.72–1.41)	0.967		
Grade (G3 vs. G2+G1)	1.37 (0.97–1.91)	0.071		
Stage (III + IV vs. I + II)	2.14 (1.51–3.02)	<0.001	2.18 (1.54–3.08)	<0.001
TMB (high vs. low)	0.99 (0.97–1.00)	0.055		
MUC16 (mutant vs. wild)	0.65 (0.44–0.94)	0.022	0.64 (0.44–0.93)	0.018

## Data Availability

The data used to perform the analyses described herein are publicly available from TCGA and ICGC data portals.

## References

[1] Ferlay J., Colombet M., Soerjomataram I. (2021). Cancer statistics for the year 2020: an overview. *International Journal of Cancer*.

[2] Sung H., Ferlay J., Siegel R. L. (2021). Global cancer statistics 2020: GLOBOCAN estimates of incidence and mortality worldwide for 36 cancers in 185 countries. *CA: A Cancer Journal for Clinicians*.

[3] Bray F., Ferlay J., Soerjomataram I., Siegel R. L., Torre L. A., Jemal A. (2018). Global cancer statistics 2018: GLOBOCAN estimates of incidence and mortality worldwide for 36 cancers in 185 countries. *CA: A Cancer Journal for Clinicians*.

[4] Llovet J. M., Zucman-Rossi J., Pikarsky E. (2016). Hepatocellular carcinoma. *Nature Reviews Disease Primers*.

[5] Bruix J., Reig M., Sherman M. (2016). Evidence-based diagnosis, staging, and treatment of patients with hepatocellular carcinoma. *Gastroenterology*.

[6] Liu Y. C., Yeh C. T., Lin K. H. (2020). Cancer stem cell functions in hepatocellular carcinoma and comprehensive therapeutic strategies. *Cells*.

[7] Hinshaw D. C., Shevde L. A. (2019). The tumor microenvironment innately modulates cancer progression. *Cancer Research*.

[8] Rao C. V., Asch A. S., Yamada H. Y. (2017). Frequently mutated genes/pathways and genomic instability as prevention targets in liver cancer. *Carcinogenesis*.

[9] Kato S., Okamura R., Baumgartner J. M. (2018). Analysis of circulating tumor DNA and clinical correlates in patients with esophageal, gastroesophageal junction, and gastric adenocarcinoma. *Clinical Cancer Research*.

[10] Hamid A. A., Gray K. P., Shaw G. (2019). Compound genomic alterations of TP53, PTEN, and RB1 tumor suppressors in localized and metastatic prostate cancer. *European Urology*.

[11] Zhu G., Pei L., Li Y., Gou X. (2020). EP300 mutation is associated with tumor mutation burden and promotes antitumor immunity in bladder cancer patients. *Aging (Albany NY)*.

[12] Calderaro J., Ziol M., Paradis V., Zucman-Rossi J. (2019). Molecular and histological correlations in liver cancer. *Journal of Hepatology*.

[13] Zucman-Rossi J., Villanueva A., Nault J. C., Llovet J. M. (2015). Genetic landscape and biomarkers of hepatocellular carcinoma. *Gastroenterology*.

[14] Boyault S., Rickman D. S., de Reynies A. (2007). Transcriptome classification of HCC is related to gene alterations and to new therapeutic targets. *Hepatology*.

[15] Shibata T. (2021). Genomic landscape of hepatocarcinogenesis. *Journal of Human Genetics*.

[16] Chalmers Z. R., Connelly C. F., Fabrizio D. (2017). Analysis of 100,000 human cancer genomes reveals the landscape of tumor mutational burden. *Genome Medicine*.

[17] Subramanian A., Tamayo P., Mootha V. K. (2005). Gene set enrichment analysis: a knowledge-based approach for interpreting genome-wide expression profiles. *Proceedings of the National Academy of Sciences of the United States of America*.

[18] Unsal M., Kimyon Comert G., Karalok A. (2018). The preoperative serum CA125 can predict the lymph node metastasis in endometrioid-type endometrial cancer. *Ginekologia Polska*.

[19] Felder M., Kapur A., Gonzalez-Bosquet J. (2014). MUC16 (CA125): tumor biomarker to cancer therapy, a work in progress. *Molecular Cancer*.

[20] Forner A., Reig M., Bruix J. (2018). Hepatocellular carcinoma. *The Lancet*.

[21] McGranahan N., Furness A. J. S., Rosenthal R. (2016). Clonal neoantigens elicit T cell immunoreactivity and sensitivity to immune checkpoint blockade. *Science*.

[22] Zuazo M., Arasanz H., Fernández-Hinojal G. (2019). Functional systemic CD4 immunity is required for clinical responses to PD-L1/PD-1 blockade therapy. *EMBO Molecular Medicine*.

[23] Shi W., Dong L., Sun Q., Ding H., Meng J., Dai G. (2018). Follicular helper T cells promote the effector functions of CD8(+) T cells via the provision of IL-21, which is downregulated due to PD-1/PD-L1-mediated suppression in colorectal cancer. *Experimental Cell Research*.

[24] Huang Y. J., Cao Z. F., Wang J. (2021). Why MUC16 mutations lead to a better prognosis: a study based on the Cancer Genome Atlas gastric cancer cohort. *World Journal of Clinical Cases*.

[25] Das S., Batra S. K. (2015). Understanding the unique attributes of MUC16 (CA125): potential implications in targeted therapy. *Cancer Research*.

[26] Hanson R. L., Hollingsworth M. A. (2016). Functional consequences of differential O-glycosylation of MUC1, MUC4, and MUC16 (downstream effects on signaling). *Biomolecules*.

[27] Aithal A., Rauth S., Kshirsagar P. (2018). MUC16 as a novel target for cancer therapy. *Expert Opinion on Therapeutic Targets*.

[28] Jiang K., Tan E., Sayegh Z., Centeno B., Malafa M., Coppola D. (2017). Cancer antigen 125 (CA125, MUC16) protein expression in the diagnosis and progression of pancreatic ductal adenocarcinoma. *Applied Immunohistochemistry & Molecular Morphology*.

[29] Chan T. A., Wolchok J. D., Snyder A. (2015). Genetic basis for clinical response to CTLA-4 blockade in melanoma. *New England Journal of Medicine*.

[30] Van Allen E. M., Miao D., Schilling B. (2015). Genomic correlates of response to CTLA-4 blockade in metastatic melanoma. *Science*.

[31] Sharabi A., Kim S. S., Kato S. (2017). Exceptional response to nivolumab and stereotactic body radiation therapy (SBRT) in neuroendocrine cervical carcinoma with high tumor mutational burden: management considerations from the center for personalized cancer therapy at UC san diego moores cancer center. *The Oncologist*.

[32] Domingo E., Camps C., Kaisaki P. J. (2018). Mutation burden and other molecular markers of prognosis in colorectal cancer treated with curative intent: results from the QUASAR 2 clinical trial and an Australian community-based series. *The Lancet Gastroenterology & Hepatology*.

[33] Huang Y., Huang X., Zeng J., Lin J. (2021). Knockdown of MUC16 (CA125) enhances the migration and invasion of hepatocellular carcinoma cells. *Frontiers in Oncology*.

[34] Bryceson Y. T., March M. E., Ljunggren H. G., Long E. O. (2006). Synergy among receptors on resting NK cells for the activation of natural cytotoxicity and cytokine secretion. *Blood*.

[35] Dianat-Moghadam H., Rokni M., Marofi F. (2018). Natural killer cell-based immunotherapy: from transplantation toward targeting cancer stem cells. *Expert Opinion on Biological Therapy*.

